RETRACTED

# The Dissemination and Evaluation of Campus Ideological and Political Public Opinion Based on Internet of Things Monitoring

**DOI:** 10.1155/2022/8294613

**Published:** 2022-06-14

**Authors:** Xiao Xu, Bei Sun

**Affiliations:** ^1^School of International Communication, Communication University of China, Nanjing 211172, China; ^2^School of E-Sports, Communication University of China, Nanjing 211172, China

## Abstract

With the advent of the information age, the rapid development of Internet of Things technology makes monitoring methods more flexible and changeable. As an intelligent application, the development of the Internet of Things brings convenience to public opinion monitoring. However, at present, due to the high price of transmission equipment, inconvenient maintenance, information delay, and other unfavorable conditions, real-time and controllable public opinion monitoring cannot be carried out on a large scale, and there are still many deficiencies in campus ideological and political public opinion monitoring. We found an effective transmission method, explored the network energy saving, dig deep into the transmission function of the signal system, and reduced the interference and mutual influence of various transmission accessories. In the application of the Internet of Things, the network public opinion is remotely monitored, the campus public opinion information is mastered, and its dissemination and development orientation are controlled. The exploration and research of online public opinion monitoring are in line with the goal of smart campus, and its theoretical development is constantly enriched.

## 1. Introduction

The Internet of Things is an emerging information technology revolution [1–5]. As an intelligent application, it has become an extremely important application field. It is an extremely effective tool for monitoring systems [6–9]. Its popularity is increasing year by year, so it is more familiar to the public. The concept of smart campus has gradually gained popularity in recent years [10–12]. It is of great practical significance for ideological and political education to grasp this trend and use the Internet of Things to carry out ideological education work. With the continuous upgrading and expansion of Internet of Things technology, we can realize real-time network remote monitoring. To better meet the needs of campus ideological and political public opinion monitoring [13], public opinion supervision is crucial to campus stability [14, 15]. We use corresponding research methods to improve the supervision of public opinion, conduct real-time mastery and supervision of campus public opinion, and manage and guide it accordingly. The development and application of ideological and political education functions through the development of corresponding modules on the network and the continuous improvement of the functional application of the Internet of Things platform are the embodiment of the comprehensive implementation of the smart campus. The exponential development of Internet platforms has greatly increased the number of online public opinions. In today's information age, the masses have considerable freedom of speech on the Internet, which makes the overall controllability of public opinion information poor. It is necessary to increase the development of public opinion monitoring tools.

RETRACTED

## 2. Overall Design of Campus Public Opinion Dissemination

In the dissemination of campus public opinion information, the dissemination of ideological and political public opinion is one of the important aspects. We need to complete these tasks: the construction of the campus Internet of Things site, the construction of the energy cycle development system, and the construction of the public opinion monitoring website. Finally, the application of monitoring model to perfect the network environment is established.

When the Internet of Things technology is applied to the construction of smart campuses, it is necessary to fully exploit and utilize the characteristics of the Internet of Things. It makes the task of campus information management in the data age more convenient and effective and can better control the development of public opinion and make it truly effective. The optimization and upgrading of the monitoring function of the Internet of Things conform to the trend of the times and meet the goal of building a smart campus, so that the management and control of campus public opinion can be truly improved.

There are three parts in the campus public opinion dissemination system. One is the monitoring system, including wireless transmission, core control. and sensing operation, which is the core application of the entire system. The second is the appropriate addition of the energy supply system, including the reasonable conversion of natural energy, which can effectively improve the efficiency of energy utilization. The last is the web page display system, which can record and call monitoring data, including time data and location data. The overall design block diagram of campus public opinion dissemination is shown in Figure 1.

### 2.1. Text Analysis and Calculation of Public Opinion

The following is the application of the TF-IDF method. We can calculate and add vocabulary weights on the basis of the original documents and assign different weights to different words, so as to achieve the division of importance. When a word appears more than average, it can be considered representative, and we perform TF-IDF assignment operation on it. This can make the entire corpus weighted, making it easier to judge the orientation of campus public opinion. This formula can be converted into document feature values for operation when the number of occurrences of words in the article is too large. Specifically, it is a weight addition and subtraction operation for dividing the importance level. The formula for calculating the TF value is as follows:

(1) $$\begin{array}{c} {\text{TF}}_{i,j}=\frac{n_{i,j}}{\Sigma_{k}n_{k,j}}. \end{array}$$

Among them, TF_*i*,*j*_ represents the TF value of the *i*th word of the *j*th article, *n*_*i*,*j*_ represents the frequency of the *i*th word of the *j*th article, Σ_*k*_*n*_*k*,*j*_ represents the frequency of occurrence of all words in the *j*th article, and *k* refers to the vocabulary size contained in the *j*th article. The introduction of the IDF calculation formula allows us to facilitate its calculation process, as shown below:

(2) $$\begin{array}{c} {\text{IDF}}_{i,j}=\log\frac{\left|D\right|}{1+\left|D_{t_{i}}\right|}. \end{array}$$

IDF_*i*,*j*_ can be specific to the IDF value of the *i*th word in the *j*th article, |*D*| represents the total number of text data, and |*D*_*t*_*i*__| represents the text number of *t*_*i*_.

RETRACTED

The overall calculation formula of the TF-IDF value is as follows:

(3) $$\begin{array}{c} \text{TF}-{\text{IDF}}_{i,j}={\text{TF}}_{i,j}\times {\text{IDF}}_{i,j}. \end{array}$$

After a large number of TF weight operations [16], extract basic emotional information from text information, so that we can understand the general orientation of public opinion and better study its control methods. Public opinion information is the expression and expression of people's emotions, reflecting the needs of the social masses. The orientation of public opinion information in today's society will cause huge social repercussions, so it is very important to carry out its monitoring work. Public discourse text information is an important aspect, and more attention should be paid to text sentiment analysis.

Naive Bayes is a hypothetical concept [17]. First, assume that the conditions are established, so that the joint behavior turns to differentiation, then gradually solve the probability, and finally apply the conditional probability to calculate.

After multiplying the probabilities, add the maximum likelihood value to solve

(4) $$\begin{array}{c} \text{PX}=x，Y=C_{k}=\text{PY}=C_{k}P\left(X=x|Y=C_{k}\right),\\ \text{PY}=C_{k}=\frac{\text{count}\left(Y=C_{k}\right)}{N}. \end{array}$$

The prior probability is represented by PY=*C*_*k*_. The maximum likelihood value proposed above also speaks of it. Usually the value of *x* is not easy to determine, which brings great difficulty to our calculation, so we have to carry out what-if analysis and use conditional independence and likelihood value to perform calculation operations:

(5) $$\begin{array}{c} P\left(X=x|Y=C_{k}\right)=P\left(X_{1}=x_{1},\ldots ,X_{n}=x_{n}|Y=C_{k}\right)\\ =\overset{n}{\underset{i=1}{\prod }}P\left(X_{i}=x_{i}|Y=C_{k}\right),\\ P\left(X_{i}=x_{i}|Y=C_{k}\right)=\frac{\text{count}\left(X_{i}=x_{i},y_{i}=c_{k}\right)}{\text{count}\left(y_{i}=c_{k}\right)}. \end{array}$$

The posterior probability is then obtained, and the *y* value is output:

(6) $$\begin{array}{c} y=\text{arg}\underset{C_{k}}{\max}\frac{P\left(X=x|Y=C_{k}\right)\text{PY}=C_{k}}{P\left(X=x\right)}. \end{array}$$

We can finally get the calculation formula of the classification prediction function by simple conversion:

(7) $$\begin{array}{c} y=\text{arg}\underset{C_{k}}{\max}\text{PY}=C_{k}\prod_{i=0}^{n}P\left(X_{i}=x_{i}|Y=C_{k}\right). \end{array}$$

After the above calculation is carried out, the text sentiment analysis value can be obtained. Then, take corresponding measures to guide public opinion information to avoid unnecessary losses.

RETRACTED

### 2.2. Storage and Operation of Information

Sentiment analysis work is very important [15, 18–21]. In the following, a series of refinement operations are performed on the public opinion text information, and the lexical sentiment weights are arranged for the text data. Through keyword search, public opinion overview and early warning operations can be performed, and crawler and training parameters can be appropriately added to store and maintain public opinion data. Its design can be drawn from Figure 2:

Because people's words and deeds on the Internet are relatively free [22–24], the speed of dissemination of public opinion information has reached an unimaginable level, and the huge vocabulary increases the difficulty of its storage. For the main body of teachers and students, network tools are used more frequently, so the task of storing public opinions on campus is more difficult. We recommend using MySQL database technology. It has the characteristics of low overhead, high efficiency, and fast speed. It can run in many environments and has good performance in different scenarios. The data hierarchy is interconnected. The differentiated operation of the monitoring system is realized through Mange management, and it also has comprehensive operation monitoring of sessions, threads, and memory. Then, connect to the database protocol communication layer data and implement SQL parsing and optimization operations through the JDBC driver. The classification structure of MySQL database is shown in Figure 3.

RETRACTED

Among them, the MySQL statement has the following advantages: MySQL statement has a good shareability, can share and exchange campus public opinion, and adapt to such a huge network public opinion system on campus. MySQL occupies less memory resources, which can facilitate our later cleaning and maintenance work, and we can run operations with less investment. The MySQL language is easy to use, is open source, and has a wealth of applicable platforms, which is convenient for campus personnel to use.

For the data set stored in the database, its reserves are quite huge. We require most of the data to be empty and only extract a small number of clearly representative data as representatives to represent the overall attributes, so as to achieve high efficiency. To identify and analyze public opinion information, we add the model evaluation analysis system to it and propose the precision rate *P*, recall rate *r*, *F*_1_, and so on. The following calculated values can be obtained through matrix operations:

(8) $$\begin{array}{c} P=\frac{\text{TP}}{\text{TP}+\text{FP}},\\ r=\frac{\text{TP}}{\text{TP}+\text{FN}},\\ F_{1}=\frac{2\text{TP}}{2\text{TP}+\text{FP}+\text{FN}},\\ \text{acc}=\frac{\text{TP}+\text{TN}}{\text{TP}+\text{FP}+\text{TN}+\text{FN}}. \end{array}$$

*P* is the overall analysis result of the predictive model, and *r* is the positive scale of the data. The *F*_1_ value represents the average value of the reciprocal, and acc is the accuracy of the data, which is the proportion of all data. After the abovementioned data storage analysis, the orientation of campus public opinion can be clearly drawn, so that we can conduct more accurate and precise guidance and facilitate the direction of public opinion.

## 3. Model Structure Optimization

### 3.1. Improvements in Energy Delivery

The power generation efficiency of traditional energy is extremely low, so we have carried out related transformations. The inverter, controller, converter, and battery have been properly adjusted, and the effect has improved. The energy initially flows to the controller and then splits into two to the inverter and battery. The inverter mainly supplies power to the equipment, and the battery stores the backup power. The specific implementation is shown in Figure 4.

### 3.2. Upgrade of Information Extraction

Generally speaking, the system of public opinion monitoring can be divided into front and rear ends. In the front-end operation, we mainly perform login options, which can roughly preview the public opinion content, watch the ranking of popular topics, search for keywords, etc., which is the main tool for understanding public opinion information. In terms of the back-end, we sequentially carry out the process of data collection, storage, extraction, and analysis and collect statistics on the collected information, so as to achieve effective monitoring of public opinion information. Its system structure diagram is roughly as shown in Figure 5.

RETRACTED

Sentiment analysis of text is extremely important. It is worth emphasizing that we individually revamp and optimize the text sentiment analysis work. We introduce the CNN-BILSTM-ATT sentiment classification model. The CNN neural network has great advantages in capturing information in local areas and can perform analysis operations on high-latitude data. Since the object of our processing is the extremely large campus public opinion information group, it is easy to cause data missing when the CNN pooling layer performs data extraction and analysis on it. RNN has the ability of time processing and can effectively complete some difficult problems in time processing. But, at the same time, when RNN encounters such huge data information, its processing ability is also poor. LSTM has a certain ability to forget data, which is extremely important for text work with a huge amount of information. The forgetting ability of LSTM allows us to exclude those neutral words, or words that are not very helpful for analysis. Finally, combining the respective advantages of these models, we concluded that the CNN-BILSTM model can effectively solve this problem and greatly improve the accuracy of data sentiment analysis. Its comprehensive structure is shown in Figure 6.

Introduce the model, adding three gates. The calculations are as follows, each responsible for forgetting filtering, transmitting information, and outputting data. The calculation is as follows:

(9) $$\begin{array}{c} f_{t}=\sigma \left(w_{f}\cdot \left[h\left(t-1\right)\right],x\left(t\right)\right]+b_{f},\\ i_{t}=\sigma \left(w_{i}\cdot \left[h\left(t-1\right)\right],x\left(t\right)\right]+b_{i},\\ ∼c_{t}=\tanh\left(w_{c}\cdot \left[h\left(t-1\right)\right],x\left(t\right)\right]+b_{c},\\ c\left(t\right)=f_{t}*c\left(t-1\right)+i_{t}*∼c_{t},\\ o_{t}=\sigma \left(w_{o}\cdot \left[h\left(t-1\right)\right],x\left(t\right)\right]+b_{o},\\ h_{t}=o_{t}*\;\tanh\left[c\left(t\right)\right]. \end{array}$$

Sequence detection of convolutional kernels is performed in the convolutional layers of the model. We set this value to *m* and calculate as follows:

(10) $$\begin{array}{c} k_{i}=\tanh\left(u_{i}*w^{\prime }+b\right). \end{array}$$

Among them, *u*_*i*_ represents the convolution kernel, and *w*′=[*w*_*i*_, *w*_*i*+1_ ⋯ *w*_*i*+*m*−1_] is a continuous *m* vocabulary vector.

RETRACTED

The output of feature vector calculation at time *t* is *O*_*t*_^*f*^, *O*_*t*_^*b*^. Then, *V*_*t*_ is calculated as follows:

(11) $$\begin{array}{c} V_{t}=O_{t}^{f}+O_{t}^{b}. \end{array}$$

Assign weights to the BILSTM layer to obtain the target weights, which are calculated as follows:

(12) $$\begin{array}{c} U_{t}=\tanh\left(v_{t}\right) \end{array}$$

The final SOFTMAX function can obtain the vector *P*_*t*_ after probabilistic operation and then calculate the weighted average to complete the calculation of each part. The relevant calculations are as follows:

(13) $$\begin{array}{c} P_{t}=\frac{\text{exp}\left(U_{t}\right)}{\sum_{t=1}^{m}\text{exp}\left(U_{t}\right)},\\ a_{t}=\sum_{t=1}^{m}P_{t}\cdot V_{t}. \end{array}$$

### 3.3. Optimization of Data Storage

In the overall framework structure of data storage applications, we are mainly dividing it into the following layers, which are user layer, application management layer, application platform support layer, application service layer, and application device layer.

The user layer mainly manages the user's data information. In the application management layer, the system settings, database, and website modules of public opinion can be applied for hierarchical data management. Subsequently, the development of multiplatform systems provides better system support capabilities. The series of platforms mainly include data acquisition and analysis and communication interfaces. Finally, it comes to the service layer, which is the application for the public, including SMS service, pop-up information service, and report download service. Its overall frame structure is shown in Figure 7.

This figure depicts the comprehensive framework of the data storage application and its overall architecture. It can be seen from the figure that the application device serves as the underlying device and has the main objects of the service on it, including short messages, information, and other content. The support layer is its core processing layer, which provides the processing work of information technology. The mutual cooperation of each application layer can finally realize the effective operation of data storage.

When it comes to data storage work, the first thing that comes to our mind is the extremely large number of chaotic information elements. In the face of these massive data information, it is very difficult for us to extract and analyze valuable factors, but we still have some. The approach makes it less complicated to sift through the data for analysis. The RBF neural structure diagram allows us to understand the principle of its data extraction. Its organizational structure is roughly as shown in Figure 8.


(14) $$\begin{array}{c} G\left(X,c_{j}\right)=e^{1/2\sigma_{j}^{2}x-c_{j}{}^{2}},\\ y=\sum_{j=1}^{m}\left(G\left(x,c_{j}\right)\times w_{j}\right). \end{array}$$

In this formula, *m* is the unit number of hidden neuron *G*, the output is *Y*, and the input is *X*. *c*_*j*_ and *σ*_*j*_ are the length and width data in the hidden layer.

(15) $$\begin{array}{c} \text{Loss}=\frac{1}{2}{\left(\hat{y}-y\right)}^{2},\\ c_{j}=c_{j}-a\frac{\partial \text{Loss}}{\partial c_{j}}=c_{j}+a\frac{w_{j}}{\sigma_{j}^{2}}\left(\hat{y}-y\right)G\left(x,c_{j}\right)\left(x-c_{j}\right),\\ \sigma_{j}=\sigma_{j}-a\frac{\partial \text{Loss}}{\partial \sigma_{j}}=\sigma_{j}+a\frac{w_{j}}{\sigma_{j}^{3}}\left(\hat{y}-y\right)G\left(x,c_{j}\right)x-c_{j}{}^{2},\\ w_{j}=w_{j}-a\frac{\partial \text{Loss}}{\partial w_{j}}=w_{j}+a\left(\hat{y}-y\right)G\left(x,c_{j}\right), \end{array}$$

where $\hat{y}$ represents the real result, *y* is the final result, and *a* is the learning rate. The RBF neural network data is continuously learned and trained to improve the learning accuracy of data analysis and speed up the learning efficiency on the basis of the machine memory ability. In continuous learning and training, find the best oscillation range. In this way, the maximum learning accuracy is obtained and the most accurate data analysis results are obtained.

RETRACTED

## 4. Experimental Simulation

### 4.1. Experimental Scheme

At the end of the experiment, we conduct a comparative analysis of the algorithm to verify its practical effect. Research campus public opinion information is the analysis object of the monitoring model. We compare multiple sets of data and obtain corresponding results by statistics on the efficiency of text sentiment analysis, the amount of text information analysis, and the delay in time transmission. The specific plans are as follows:

  Option 1: TF-IDF method and MySQL database screening for public opinion data analysis
  Option 2: TF-IDF method combined with MySQL database to provide energy-optimized public opinion data analysis
  Option 3: TF-IDF method, public opinion data analysis after introducing CNN-BILSTM-ATT sentiment classification model into MySQL database
  Scheme 1: TF-IDF method, MySQL database combined with CNN-BILSTM-ATT sentiment classification model and RBF neural network to analyze the final public opinion information

### 4.2. Public Opinion Analysis and Comparison

Through the design of the above four schemes, we respectively set up a public opinion sentiment analysis experiment with the number of public opinion data information as 200, 500, 1000, and 3000 as the basic amount of data 3000. The results can clearly see the strength of each scheme for sentiment analysis. The specific comparison is shown in Figure 9.

RETRACTED

In the following, we will study the time analysis efficiency of various schemes. In the specified unit time, the algorithm analysis amount of schemes 1–4 will be counted, respectively. After comparison, it can be clearly seen that the optimization of scheme 1 has improved significantly. Especially after 4 minutes, the pros and cons of the algorithm are more obvious. The amount of data analysis of scheme 1 is significantly higher than that of other categories. It can be seen more clearly the data analysis ability of our optimized model. The quantitative analysis comparison is shown in Figure 10.

Time efficiency is an important performance metric in any algorithm. The amount of data transmission per unit time of the algorithm is one of the important manifestations. It can be clearly seen from the time delay comparison analysis chart of the four algorithms that the time loss of scheme 1 is significantly lower than that of other algorithms. From left to right, the amount of data selected by the time delay is 100, 300, 500, and 1000, and the specific time loss comparison is shown in Figure 11.

Next, we use the fixed length of public opinion texts as a statistic to explore the efficiency ratio of each scheme to show the distribution of the highest efficiency. Not surprisingly, scheme 1 is the least efficient, while scheme 1 accounts for more than half of the total analysis efficiency, which is equivalent to the sum of the other three algorithms. The specific efficiency distribution is shown in Figure 12.

In the division of market satisfaction based on a fixed number of people, Schemes 1–4 have achieved different results. In the comparative analysis chart, the superiority of option 4 can be clearly seen, and its satisfaction level even reaches about 95%, which clearly shows the public's recognition of it, specifically as shown in Figure 13.

### 4.3. Analysis and Evaluation of Public Opinion

Among the numerous information data, we finally obtained two forms through the algorithm collection and analysis, one is the relevant information introduction of the search, and the other is the user's information description. In the search information, we can clearly know the user ID, the completion time of the search, the number of likes and retweets, etc., and even the text content of the search relevance. In the user specific information, we can learn some content, such as name and age. The acquisition of the following information data enables us to quickly understand the direction of public opinion dissemination, which brings great convenience to the detection work and more effectively controls the development of public opinion. The details are shown in Tables 1 and 2.

RETRACTED

In order to further verify the practical application ability of the public opinion data improvement model, we conducted a comprehensive data collection and analysis experiment, using the optimal algorithm for experimental operation, and running the algorithm under the condition that the optimal parameters are set as the benchmark to obtain the data in Table 3. It can be seen that the accuracy of the analysis of public opinion information in this experiment is very high, with an average of more than 95%. The specific situation is as follows:

## 5. Conclusion

In today's network information age, with the continuous popularization of network use, the amount of public opinion information is huge, and its management and monitoring are increasingly important. It is necessary to supervise and control the sensitive information and guide the trend of public opinion reasonably. These are all we need to do. In campus public opinion, topics with political tendencies are particularly important. If some negative emotions are added to them, it may affect the public's value orientation and bring about serious social problems. We must take measures to control them. This paper uses TF-IDF method to add and subtract weights and MySQL database and CNN-BILSTM-ATT sentiment classification model, combined with RBF neural network, to extract and analyze public opinion texts. Then, add a text sentiment analysis model for algorithm analysis. Implement the search and supervision of user information, and achieve a comprehensive upgrade of the accuracy of public opinion monitoring. It effectively avoids the serious problems caused by bad public opinion information. After a series of optimizations, it is more in line with the needs of campus public opinion monitoring. The monitoring of campus public opinion is of great practical significance. This paper mainly conducts exploration and research on public opinion text information and does not involve media such as pictures, voice, and video. Since these are also important aspects that reflect the trend of public opinion of the masses, comprehensive consideration of these will also be added in future research to expand public opinion monitoring, depth and width. Through the development of network modules, we improve its functions and continuously promote the construction of smart campuses.

## Figures and Tables

**Figure 1:** Overall block diagram of campus public opinion communication design.

**Figure 2:** Analysis of public opinion text data.

RETRACTED

**Figure 3:** MySQL database implementation flow chart.

**Figure 4:** Hardware allocation process of energy supply structure.

**Figure 5:** Structure diagram of public opinion monitoring system.

**Figure 6:** CNN-BILSTM model structure diagram.

**Figure 7:** Overall framework of data storage applications.

**Figure 8:** RBF neural network diagram.

**Figure 9:** Comparison of public opinion sentiment analysis.

**Figure 10:** Unit time analysis and comparison chart.

**Figure 11:** Unit data time delay diagram.

**Figure 12:** Efficiency ratio of text length analysis.

**Figure 13:** Market satisfaction.

**Table 1:** Search information table.

Id	Primary key
User-id	User ID
Like-num	Likes
Retweet-num	Number of retweets
Keyword	Search keyword
Create-time	First acquisition time
Update-time	Last acquisition time
Target	Search title
Href	Search link
Click	Have hits
Rank	Heat
Tag	Is it relevant

**Table 2:** User information table.

Field name	Explain
Id	Primary key
Nickname	Username
Gender	User gender
Location	User location
Description	User profile
Keyword	User search content
Talent	User credit
Work	User work information

**Table 3:** Comprehensive data analysis table.

Data set	Correct rate (%)	Recall (%)
Cluster1	91.02	89.56
Cluster2	94.57	92.65
Cluster3	92.09	96.77
Cluster4	93.25	83.59
Cluster5	98.57	96.64
Cluster6	95.65	91.56

## Data Availability

The experimental data used to support the findings of this study are available from the corresponding author upon request.
